# Treatment of Large and Complicated Scalp Defects with Free Flap Transfer

This article has been retracted.

**DOI:** 10.1155/2020/2748219

**Published:** 2020-01-10

**Authors:** Fanfan Chen, Hongbin Ju, Anfei Huang, Yongjun Yi, Yongfu Cao, Wei Xie, Xinliang Wang, Guo Fu

**Affiliations:** ^1^Department of Neurosurgery, The Second People's Hospital of Shenzhen, Shenzhen, Guangdong 518035, China; ^2^Department of Orthopaedics, Guangzhou First People's Hospital, Guangzhou, Guangdong 510180, China; ^3^Department of Spine and Orthopedic Trauma, The First Affiliated Hospital of Jinan University, Guangzhou, Guangdong 510630, China

## Abstract

**Background:**

Large scalp defects, especially those complicated by calvarial defects, titanium mesh exposure, or cerebrospinal fluid (CSF) leak, pose a challenge for the neurosurgeon and plastic surgeon. Here, we describe our experience of reconstructing the complex scalp defect with free flap transfer.

**Methods:**

From October 2012 to September 2017, 8 patients underwent free flap transfer for the reconstruction of the scalp or complicated scalp and calvarial defects. Five patients presented with scalp tumor and the other 3 patients with scalp necrosis or ulceration (2 patients with titanium plate exposure). Seven anterolateral thigh flaps and one radial forearm flap were harvested and employed. The clinical data, including defect characteristics, flap type, complications, and outcomes, were recorded and analyzed.

**Results:**

Five patients were pathologically diagnosed with malignant tumor, and 3 of them were given further radiotherapy. For the 2 patients with exposure of titanium plate, no titanium plate was removed. For the patient with scalp necrosis after decompressive craniectomy accompanied by CSF leakage, the CSF leak was stopped after reconstruction. The size of the flaps ranged from 3 to 14 cm in width and 4 to 18 cm in length. No flap failure occurred in these cases. From follow-up to the present, no ulceration or necrosis occurred.

**Conclusions:**

Free flap transfer is an ideal method for the reconstruction of large, complicated scalp defects with a one-stage operation. The anterolateral thigh flap is favored because of its durability, adjustability, water tightness, and infection prevention.

## 1. Introduction

Large scalp defects are usually secondary to a variety of diseases, such as tumor resection, trauma, infection, and congenital lesions [1, 2]. Reconstruction of the defects should take a comprehensive consideration of size, location, radiation history, and potential for hairline distortion [3]. When the scalp defect is accompanied by a calvarial or dural defect, for example, from scalp and skull bone excision due to tumor invasion, scalp necrosis after decompression surgery, scalp atrophy, or necrosis after titanium plate implant, more related factors affect the therapeutic strategy. The soft tissue coverage of the defect areas, maintaining the enclosed space for the intracranial contents, sealing the leakage of the cerebrospinal fluid (CSF), and endurance to radiation are all common concerns. This is a challenge for neurosurgeons and plastic surgeons and requires close collaboration between them.

The reconstructive ladder of scalp defects includes primary closure, split-thickness skin graft, local flap, rotated local flap and skin graft, and free flaps. For the large size of soft tissue defects on the scalp, reconstruction with local flap is restricted to the inelasticity and rotation angle. Free flap is the only available method to cover the defect. Currently, there is a lack of consensus regarding which procedure is superior in large and complicated scalp reconstruction. In this retrospective study, we present our experience with the reconstruction of scalp defects with free flap transfer. The patients and defect conditions, reconstructive options, advantages of free flap transfer, and complications are described and discussed.

## 2. Materials and Methods

### 2.1. Patient Data

This retrospective study was approved by the ethics committee of Guangzhou First People's Hospital. All the patients provided written informed consent for the use and publication of data for research purposes. Eight patients with scalp defect underwent free flap reconstruction in Guangzhou First People's Hospital from October 2012 to September 2017 (Table 1). Four men and 4 women were enrolled in this research. The patients' ages ranged from 27 to 70 years (mean, 50 years; median, 51 years). Five patients were diagnosed with scalp tumor (Figures 1(a) and 2(a)). Two patients presented with ulcer of the scalp with titanium plate exposure (Figure 2(d)). The remaining 1 patient had scalp necrosis after decompressive craniectomy accompanied by CSF leakage. The area of the defect was located in the forehead region (1 case), the frontoparietal region (1 case), the frontal region (1 case), the lateral occipital region (1 case), the parietal to occipital region (2 cases), and the temporal region (2 cases).

### 2.2. Surgical Technique

All the patients received a routine preoperative examination. No signs of general or local infection were found. For the patients with scalp malignancies, tumor infiltration of the periosteum or skull was evaluated, and excision of the skull bone was performed accordingly. For the cases of titanium mesh exposure or scalp necrosis, thorough debridement and excision of the nonvascularized tissue were accomplished. All the reconstructive procedures were performed by the same surgeon. An anterolateral thigh (ALT) fasciocutaneous flap was employed in 7 patients (Figures 2(b) and 2(c)) and a radial forearm flap was used in 1 patient (Figures 2(e) and 2(f)). The facial artery and facial vein were anastomosed with the vessel pedicle of the flap passing through the subcutaneous tunnel in 6 cases. Branches of the external carotid artery and superficial temporal artery were used as the recipient artery in 1 case. The muscular component was not harvested in most cases. When elimination of “dead space” was necessary, proper bulk of muscle was preserved (Figure 1(c), arrow). The superficial temporal artery and vein were used in 1 case. The follow-up period was 3 to 36 months.

## 3. Results

The pathology of 5 cases diagnosed as malignant scalp tumor included squamous cell carcinoma (2 cases), basal cell carcinoma (2 cases), and adenocarcinoma (1 case). Two patients underwent partial calvarial excision and titanium mesh implantation, as the skull was invaded by the tumor. Three patients (including the 2 patients with titanium mesh) were treated with further radiotherapy, and the other 2 patients refused radiotherapy. The ALT flaps were used in 7 patients, and the radial forearm flap was employed in 1 case. The size of the flaps ranged from 3 to 14 cm in width and 4 to 18 cm in length. Fasciocutaneous flaps were harvested for reconstruction. The remaining 3 patients, 2 patients with titanium mesh exposure and 1 patient with scalp necrosis and CSF leak after decompressive craniectomy (Figure 3(a)), were reconstructed with fasciocutaneous flap as well. The patients were followed-up from 3 to 36 months. No major complications such as flap failure, vascular pedicle thrombosis, necrosis, or ulceration after radiation occurred. The survival rate of the flaps was 100%. Wound dehiscence was found in 2 cases, and the incisions healed after local resuturing. The patient with CSF leak had resolution of the leak after flap reconstruction. No secondary infection occurred. Neither CSF leakage nor extradural effusion was found. The donor site defects of 6 patients were primarily closed, and 2 patients received split-thickness skin grafting.

### 3.1. Case 1

A 62-year-old woman was diagnosed with adenocarcinoma with tumor invasion of the right mastoid and occiput (Figure 1(a)). An extensive excision of the tumor, underlying the skull bone and regional lymph node, was performed with titanium mesh implantation (Figure 1(b)). An ALT flap (13 × 15 cm) was used to cover the scalp defect (Figures 1(c) and 1(d)). The patient subsequently underwent radiotherapy, and within the 12-month follow-up period, no tumor relapse or flap abnormality were found (Figure 1(e)).

### 3.2. Case 2

A 54-year-old woman in a persistent vegetative state had scalp necrosis at the incision of a previous decompressive surgery (Figure 3(a)). A CSF leak was found along the lesion, but no general or local infection was found. A thorough debridement of the lesion was performed before an ALT flap (7 × 12 cm) was used to reconstruct the defect (Figure 3(b)). The CSF lead was stopped postoperatively, and the condition of the flap was uneventful in the 9-month follow-up period (Figure 3(c)).

## 4. Discussion

Large full-thickness scalp defects are a refractory problem for treatment due to the low elasticity of the scalp. Primary closure or local flap transposition is insufficient for reconstruction of large defects or is prone to subsequent atrophy and ulceration due to improper tension. The detailed conditions of each patient should be taken into consideration [3]. For example, the condition of the adjacent scalp of the defect, concomitant scalp and calvarial defects, scalp defects with previous foreign material implantation, the possibility of subsequent radiotherapy, and the general condition of the patient are all closely related to the reconstructive choice. The 2 cases presented in detail were especially difficult. Of the 5 patients diagnosed with scalp tumor (including squamous cell carcinoma, basal cell carcinoma, adenocarcinoma, and dermatosarcoma), 3 of them were treated with further radiotherapy (Figures 2(a)–2(c)), and 2 of these 3 patients underwent titanium plate implantation, as the skull was invaded by the tumor. The ideal reconstructive method should be enough to cover the defect with proper tension, require the least operative time, and be durable for any subsequent radiotherapy. The remaining 3 patients had brain hemorrhage or brain injury followed by at least two cranial surgeries before the necrosis or ulceration of the scalp. Two patients presented with exposure of the titanium mesh (Figure 2(d)). For the patient who had not had a cranioplasty, CSF leakage occurred. This particular patient was in a persistent vegetative state and had malnutrition. Fortunately, no intracranial infection was observed in this patient. Based on all these adverse factors, reconstructive procedures must be well vascularized, watertight, and able to prevent infection [4]. Although small forehead defects can be effectively repaired by reversed temporal island flap [5], the condition of surrounding scalp, temporalis, and superficial temporal artery should be in good condition. Our patient bearing the forehead scalp defect had previously experienced times of surgeries which resulted in a vulnerable blood supply and poor condition of nearby scalp (Figure 2(d)). Under this situation, free flap transfer offered a more stable coverage.

The microsurgical free flap transfer for the reconstruction of the scalp has developed ever since it was first performed by McLean and Buncke [6]. In its first application, an omental flap was used to reconstruct a large scalp defect. Although the omental flap was not accepted by later surgeons because of the creation of the laparotomy, the concept of free tissue transfer impressed surgeons. Various donor sites for free flap transfer were achieved and described in articles, including the latissimus dorsi musculocutaneous flap, the radial forearm flap, and the rectus abdominis myocutaneous flap, to name a few [7–10]. The latissimus dorsi musculocutaneous flap and radial forearm flap were popularly used before 2000, and the ALT was more frequently adopted later [11]. Skin graft and posture change during surgery are the disadvantages of the latissimus dorsi flap. As for the radial forearm flap, inadequate size for large defects is the major limitation. The rectus abdominis muscle flap was a commonly used flap, whereas donor site complications are a major shortcoming. The ALT flap has gained more attention for tissue defect reconstruction after the description of Song et al. [12], after which this type of flap was technically refined and advocated by surgeons and widely used for reconstructive surgeries [13–16]. The advantages of the ALT flap include no requirement of position change during surgery, a long vascular pedicle with suitable size for microsurgical anastomosis, enough wide and long cutaneous area, usually direct closure of the donor-site defect, and acceptable morbidity. Moreover, the adequately vascularized fascia component of the flap is helpful to prevent CSF leakage and secondary infection [17].

Nowadays, the reconstruction of scalp defects still remains challenging. Limited sources of local or regional flaps due to the inelasticity of the scalp restrict the practice of primary closure or local flap transposition in most situations of large scalp defects. Moreover, the compromised blood supply and quality of the adjacent scalp affected by previous surgeries limit the application of a local flap. When closing defects accompanied by titanium exposure or CSF leak, multiple-stage procedures (e.g., removing the titanium mesh and replacing it after wound healing) increase the suffering of the patient. Based on all these factors and our experience, free flap transfer is the most reliable and preferred choice in a one-stage operation.

In our study, the ALT flap was chosen in 7 of 8 cases. One patient with small defects was given a radial forearm flap (Figure 2(e) and 2(f)). The relative thinness and adjustable thickness compared with the dorsi latissimus flap are important merits that make the ALT flap adaptable for different defect depth, either a superficial scalp defect due to cranioplasty or a relatively deep defect without cranioplasty. As mentioned previously, avoiding postoperative infection from foreign matter and CSF leak are also major concerns. The ALT flap offers adequate vascularization both for the dura and the scalp, which is more effective for the prevention of infection than skin grafts or local flaps. The watertight fascia layer of the ALT fasciocutaneous flap is an ideal autologous material for sealing the CSF leak [4, 18, 19].

The complication of free flap transposition includes flap failure, vascular pedicle thrombosis, donor site hematoma, calvarial oseteomyelitis, and wound dehiscence. Of our patients, no flap failure or vascular pedicle thrombosis occurred. In addition, no intracranial complications or CSF leak occurred postoperatively. Wound dehiscence occurred in 2 patients, and the wounds healed after local revision.

The limitations of this study are that the sample size is relatively small and the experience results from a single medical center. A further multicenter study may offer more powerful evidence and experience of the reconstruction of the complex scalp defects.

## 5. Conclusions

In summary, free tissue transfer is an excellent method for reconstruction of scalp defects, especially in complicated situations such as calvarial defects, titanium plate exposure, or CSF leakage. The ALT flap is ideal for large scalp reconstruction with the advantages of durability, adaptability, infection prevention, and watertightness.

## Figures and Tables

**Figure 1:** An anterolateral thigh (ALT) flap was adopted to reconstruct the complicated scalp defects of a 62-year-old female patient. (a) The lesion was located at right lateral occipital region. (b) A radical excision of the lesion, skull bone, and relevant lymph nodes was performed with a titanium mesh implanted. (c) An ALT flap was harvested with part of quadriceps to fill the dead space. (d) The postoperative image of the patient. (e) The patient received radiotherapy and the flap maintained scalp contour at 12-month follow-up.

**Figure 2:** Typical cases of free flap transfer in the reconstruction of the complicated scalp and calvarial defects. (a) A patient presented with giant scalp tumor and the tumor with the invaded skull bone was resected. (b) An ALT flap was adopted to reconstruct the scalp defect (a titanium mesh was used to reconstruct the skull defect). (c) The flap maintained the scalp contour with durable coverage of the defect. (d) A patient presented scalp defect and titanium exposure. The patients experienced several operations and the situation of adjacent scalp was poor. (e) A radial forearm flap was harvested for the reconstruction. (f) The vessels of the flap were anastomosed to the right superficial temporal vessels.

**Figure 3:** An ALT flap was used to reconstruct the complicated scalp and calvarial defects of a female patient after decompressive craniectomy. (a) The patient presented with scalp necrosis and cerebrospinal fluid leak. (b) An ALT flap was used to reconstruct the defect. (c) The situation of the flap at 9-month follow-up without CSF leak.

**Table 1:** Clinical data of patients.

Patient	Age	Sex	Etiology	Location	Treatment and flap	Flap size (width ∗ length, cm)	Follow-up (months)
1	27	Male	Ulcer with titanium plate exposure	Forehead	RF flap transfer	3 ∗ 4	3
2	64	Male	Malignant tumor	Parietal-occipital	ALT flap transfer	10 ∗ 12	36
3	70	Female	Malignant tumor	Frontoparietal	ALT flap transfer	7 ∗ 9	6
4	54	Male	Malignant tumor	Parietal-occipital	ALT flap transfer, titanium mesh implantation	12 ∗ 18	12
5	58	Female	Malignant tumor	lateral occipital	ALT flap transfer, titanium mesh implantation	13 ∗ 15	12
6	47	Female	Necrosis after decompressive cranioectomy, CSF leak	Temporal	ALT flap transfer	7 ∗ 12	9
7	38	Female	Ulcer with titanium plate exposure	Temporal	ALT flap transfer	9 ∗ 13	12
8	41	Male	Malignant tumor	Frontal	ALT flap transfer, titanium mesh implantation	14 ∗ 18	6

## Data Availability

The data supporting the findings of this study are available from Guangzhou First People's Hospital, but restrictions apply to the availability of these data, which were used under license for the current study and are not publicly available. However, the data are available from the authors upon reasonable request and with permission from Guangzhou First People's Hospital.

## Abbreviations

CSF: Cerebrospinal fluid
ALT: Anterolateral thigh.
